# The Dilemma of the Great Development of Rural Tourism from the Sustainable Environment Perspective

**DOI:** 10.1155/2022/7195813

**Published:** 2022-05-20

**Authors:** Qin Yang, Jian Li, Youlin Tang

**Affiliations:** ^1^School of Economics and Management, Shaoyang University, Shaoyang, Hunan 422000, China; ^2^Doctor of Philosophy in Education, Adamson University, Manila 1007, Philippines

## Abstract

Demand and motivation are powerful indicators of people's decisions and behaviors. Based on the in-depth interviews with 190 relevant stakeholders, the study found that the rural tourism industry is facing three kinds of pressures for continued growth. Under these three pressures, the rural tourism industry tends to “copy” and plunder resource-based development, which restricts the industry's sustainable growth path. Therefore, to continue the development of the rural tourism industry, we need to create a development path suitable for the sustainable development of rural tourism from three aspects: system, atmosphere construction, and market orientation.

## 1. Introduction

A recent study estimated that over 90% of country houses and resort hotels in China are losing money, which have to close their doors because they cannot support their daily operating expenses (https://googl.com). Rural tourism activities and rural tourism investment are increasing, but rural tourism industry is not growing [1]. Researchers and organizations call for solving the plight of rural tourism development and promoting high-quality development of rural tourism [2–4]. The term “high-quality development” refers to behavior diversification of development models, differentiation and development of product types, increased core competitiveness, improved service quality, enhanced radiation driving capabilities, etc. A recent report found that although rural tourism investors or rural tourism planners say they want to develop tourism sustainably, only a few of their specific practices are sustainable development behaviors (https://sohu.com). Researchers also found that there is a generation gap between rural tourism investors or rural tourism planners and rural destination residents regarding the values of sustainable development [5]. Although most rural tourism investors or rural tourism planners are aware of rural tourism development issues, they do not know how to solve them and avoid them [6, 7]. How can we minimize this gap?

What factors determine the sustainable development of rural tourism? Corresponding insights are procvided from two different assumptions of human motivational behavior. Ouellette and Wood [8] suggested that human behaviors result from habits and that past behaviors can shape current and future behaviors. One hypothesis is that the relevant stakeholders of the great development of the rural tourism industry are regarded as “economic persons” pursuing utility, and the relevant stakeholders as rational economic persons participate in rural tourism according to the principle of pursuing maximum profit; another hypothesis is rural tourism relevant stakeholders of large development are regarded as “social people” who pursue the needs of different levels. It is believed that the pursuit of relevant stakeholders should be considered from Maslow's hierarchy of needs. Being in a large development environment of rural tourism not only considers material needs but also more. It is the realization of safety needs, belongingness and love needs, esteem needs, and self-actualization needs. These two assumptions also mean that, in addition to “pursuing efficiency,” the stakeholders involved in the development of rural tourism may also be constrained by a certain policy environment and fail to achieve “fair gain.”

In this study, we use Demand Motivation Theory (DMT) as the basis of motivation theory analysis of microscopic subject behavior. The purpose of the study was two-fold: first, to discover the impact of interest demands of different stakeholders on the development of rural tourism; second, to test the main factors that inhibit the development of rural tourism.

The phenomenon that long-term unsatisfactory appeals for interests will lead to changes in the behavior of the actor and even escalation of conflicts among stakeholders [9, 10]. Maslow [11] divides human needs from low to high into five levels. Demand will be repeated and upgraded. Therefore, understanding the current interest levels of stakeholders is the key to solving the problem.

The existing literature gradually realizes the importance of two hypothetical theories explaining the participation of relevant stakeholders in rural tourism. For example, Jessica and Kathleen [12] believe that maintaining and enhancing the happiness of participating subjects are the key to break the obstacles in the development of rural tourism. Chin et al. [13] established an evaluation and development model to investigate the impact of rural tourism hardware services (infrastructure and accommodation) and software services (service scope and service characteristics) on the competitiveness of rural tourism destinations. Ghaderi et al. put forward the results of community capacity building (CCB) through semistructured interviews with relevant stakeholders to influence community residents' support for rural tourism. Lin and Wang [14] believe that government policy subsidies can attract investment from tourism enterprises and expand the scale of rural tourism. Ma and Luan [1] believe that the return on investment of enterprises will affect the direction of investment. Only by optimizing institutional arrangements and deepening the reform of enterprise systems, preventing excessive competition will undoubtedly increase the confidence of enterprises in investment and enhance the quality advantage of tourism economy. Wen and Yong [15] believe that the realization of the economic benefits of the community residents and the optimization of the ecological environment will affect the community residents' support for the development of rural tourism. Wang [16] pointed out that the key to realizing the great development of rural tourism is the centralized management of rural tourism resources and the best way is to realize the collective economic model.

## 2. Review of the Literature

### 2.1. A Great Development in Rural Tourism Sectors

A great development in sustainable mass tourism has become the emerging and desired outcome for most destinations [17]. A great development includes the following: (1) a general tendency to expand the scale of rural tourism; (2) high service quality and supply level of rural tourism; (3) more and more stakeholders are participating in rural tourism (e.g., [18, 19]). With the great development of rural tourism, there has been an increase in the negative impacts of tourism on this destination; stakeholders' conflicts continue to occur [20].

Rural tourism investors or rural tourism planners have established sustainable development plans when developing rural tourism projects, but they have not done so in practice. Researchers have also found a discrepancy between stakeholders' development knowledge, their attitudes toward the great development, and their actual rural tourism. For example, local governments, developers, and residents participating in tourism development are prone to form an asymmetrical power relationship because of their different resources [21]; therefore, the rural space under tourism development must be permeated with political relations and ideology [22]. This discrepancy is partially due to interest, as made by [9, 23], who showed that most local governments and enterprises tend to obtain short-term economic benefits through the development of tourism resources, rather than long-term sustainable development strategies. Sun et al. [24] likewise claimed that rural tourism makes the production activities of traditional rural communities mainly obtain production and living materials from the natural environment (land), increasing the goal of benefiting from the tourism industry, which will lead to changes in the internal logic of rural community residents regarding production. Other factors, such as lack of innovation, comfort, culture, and local characteristics, further contributed to the gap between knowledge and attitudes towards sustainable great development (https://Sohu.com, 2019). Moreover, an increasing number of customers prefer to stay in environmentally friendly, green development type rural tourism destination, but they also admit that doing so will involve increased convenience and cost [25]. How to bridge the gap between knowledge and attitudes toward sustainable great development is currently under much-needed investigation.

### 2.2. Stakeholders' Behavior under the Theory of Motivation

Motivation theory believes that organizations and individuals live in a certain environment, and the driving force generated by their behavior depends on the objects in the environment. The activities and reactions under this logic of behavior are logical deductions recognized by the social environment, that is, following a reasonable demand mechanism [11]. The drive here includes “social normative, value structure, and internal drive of resource element allocation that provide a guiding and practical significance for behavioral drive” [11, 26]. Therefore, the drive contains three basic elements: social norm elements, value structure elements, and resource allocation elements. They all provide three related but distinctly different supports for organizations and individuals to participate in the development of rural tourism.

### 2.3. Social Normative Elements

Social normative elements include formal rules, legal systems, and informal folk customs, customs, and morals [27]. Their impact on the behavior of organizations and individuals is to impose rules on others based on the corresponding legal and moral constraints, and it can also induce people to follow the rules by inspiring the needs that are rooted in the heart to be recognized. Therefore, following the rules is the rational basis for behavior [28].

From the research literature, it is found that social normative elements have an important role in promoting the sustainable development of rural tourism. Since 1994, the academic community has tried to study rural tourism as a special activity in sustainable tourism activities. For example, the European Union specifically proposed that rural tourism should provide policy support to rural tourism in terms of funding, policies, education, and training. The United States and Canada have advocated the sustainable development of rural tourism through methods such as propaganda and education. Font and Elgammal [29] believe that the development of rural tourism with green as the standard can not only legalize consumers' green consumption of landscapes but also dilute complex issues and regulate sustainability to reduce consumers' guilt for environmental damage, while protecting enterprises free from consumer doubt. Therefore, the following hypothesis is proposed: H1: there is a significant and positive relationship between social normative elements and their attitudes toward sustainable development of rural tourism.

### 2.4. Value Structure Elements

Zeithaml [25] proposed that perceived value is the overall utility of the product or service after weighing the benefit that stakeholders can perceive (benefit) and the cost (sacrifice) in obtaining the product or service. In recent years, scholars have constructed a variety of perceived value models. For example, for the consumer perceived value structure, Kantamneni and Coulson [30] proposed multidimensional product perceived value model that divides consumer perceived value into social value, experience value, functional value, and market value; Sheth et al. [31] proposed the consumer value model that divides consumer perception value into functional value, emotional value, social value, and cognitive value. Regarding the value structure of investment perception, Zeng and Huang [32] believe that the functional value, unique value, economic value, and experience value of return on investment affect the investment decision of supporters. Schwartz [33] proposed that values are beliefs that override any specific situation. This belief guides the selection and evaluation of behaviors and events and is related to the desired outcome state and behavior.

Therefore, the elements of the value structure will impose certain restrictions on the behavioral motivation of the organization and the individual, but if a certain force beyond the standard value structure is given, the behavioral motivation of the organization and the individual has an enabling effect.

Compared with conventional tourism development, rural tourism development has a completely different concept and development process on how to organize limited resources to develop rural tourism, especially how to view the sustainable development of rural tourism. Miller's [34] empirical research on the US tourism industry shows that conventional tourism believes that tourist satisfaction and higher industry chain spillover effects can achieve the sustainable development of tourism, while the sustainable development of rural tourism not only requires tourists to be satisfied but also relatively competitive. High economic spillovers also require environmental sustainability and the improvement of local residents' living environment, especially the impact of hiring locals and local social and cultural integration. Therefore, the following hypothesis is proposed: H2: there is a significant and positive relationship between value structure elements and their attitudes toward sustainable development of rural tourism.

### 2.5. Elements of Resource Allocation

Mankiw [35] believed that the scarcity of resources and the infiniteness of desires cause people to face trade-offs when making decisions, that is, they are faced with the problem of having to allocate resources. As the socioeconomic development reaches a certain stage, whether it is consumers or suppliers, the resources they can control are scarce. Therefore, in most situations, people will follow the endowment effect because in the decision-making process of people's balance of interests, the consideration of “harm avoidance” is far greater than the consideration of “increasing profits.”

The factors of resource allocation have a far-reaching impact on the sustainable development of rural tourism. Thaler [36] believes that people should avoid losing what they have, and it is easy to produce a “comfortable status quo” complex, and they are afraid of the loss caused by change. For example, when the government requisitions land, community residents often feel that the compensation provided by the government is too low and conflict with the government. In the development of rural tourism, in order to avoid the uncertainty caused by innovation, companies often use copying tourism products, resulting in rural. The phenomenon of tourism development is similar. Therefore, the following hypothesis is proposed: H3: there is a significant and positive relationship between resource allocation elements and their attitudes toward sustainable development of rural tourism.

## 3. Materials and Methods

### 3.1. Instruments

A quantitative research design was adopted in this study, using in-depth interviews to explore the impact of relevant stakeholders on the sustainable development of rural tourism. There are three reasons for choosing the in-depth interview method: first, how does the rural tourism industry as an emerging industry (because its development time is shorter than other industries), especially the key industries of the rural revitalization strategy, affect the “three rural” issues. We still lack in-depth understanding of the impact on participating stakeholders. The use of in-depth interviews is helpful for researchers to obtain different new explanations for unknown fields or for an apparent problem. Second, in-depth interviews are not affected by the original questionnaire framework. Through chatting, we can get a more realistic explanation of the problem, which is conducive to a deeper understanding of the problem. Third, in-depth interviews can break through the researchers' original expectations and expected conclusions, which is conducive to the discovery of new problems and broadens the horizon of research problems.

### 3.2. Sampling and Data Collection

From October 2016 to December 2018, the sample community residents, tourists, and residents of 8 villages in three provinces including Luohe and Luoyang in Henan Province, Shaoyang and Yueyang in Hunan Province, and Shaoguan and Meizhou in Guangdong Province participated in this study. Semistructured interviews were conducted by enterprises, village collective economic organizations, and relevant government officials. The interviews were conducted as one-on-one in-depth interviews. The interviews were conducted at the rural tourist destinations where the interviewees were active. The questions interviewed focused on the attitudes, viewpoints, actions, and sustainable development of rural tourism, mainly including three categories: one is the opinions and attitudes about the development of rural tourism, such as the ecological environment, economic income, life methods, resource use, and standards for measuring sustainable development; second, actions related to rural tourism development, for example, what methods should be adopted to provide corresponding tourism products for the sustainable development of rural tourism; and third, regarding the sustainable development of rural tourism such as the problems and challenges faced by sustainable development, as well as the willingness of all stakeholders for sustainable development. The research is conducted in the form of an interview group consisting of 2-3 people. After the discussion, the interview team initially drafted the interview outline, trying to break through the fixed visit framework, and used open-ended questions to understand the subjective feelings of the sample community residents, tourists, enterprises, village collective economic organizations, and relevant government officials. Because of the large differences in the interests of the interested parties of the interview and whether the interview questions need to be kept confidential, the interview will be conducted after obtaining the consent of the interviewee. In the interview process, the differences between the interviewer's customs and language, trying to describe their own true feelings or ideas and suggestions in their own language, are taken into account. The duration of the interview is not limited by time, but at least 45 minutes. After the interview, the researcher will organize the corresponding transcripts or recordings according to the interview process into text drafts. Lincoln and Guba [37] believe that, in order to obtain the most authentic content and the most effective information of in-depth interviews, attention should be paid to the saturation of information in the number of interviews and the content of interviews. That is to say, when the information obtained is repeated and there is no new content, there should be a courtesy to end the interview.

### 3.3. Data Analysis

After in-depth interviews, in order to obtain the understanding and attitudes of different stakeholders on the sustainable development of the rural tourism industry, the researchers need to record the spoken records and emotional responses of the interviews in writing. After completing the text records, through detailed reading of each record, we invite relevant experts and researchers to identify the text records. Based on this, we can infer which written records are related to the research theme and which are not related to the research theme. Based on the technical analysis of Lincoln and Guba [37] and Glaser and Strauss [38], we strictly collect samples and analyze qualitative data acquisition that confirms the sampling, assists the subsequent data collection, clearly defines the theme, determines the comprehensive level through the review, and makes a preliminary conceptual definition based on the theme and content. After the concept is determined, the next step is to encode the concept. It is determined that the information data start to be grouped into categories, that is, open coding. The relationship between each main category and the core category forms selective coding and clarify the “story line.” The data coding analysis method after the above in-depth interviews refers to that of Corley and Gioia [39], which is used to analyze the semistructured information data after the semistructured interviews, which are used to analyze the ambiguity and change of the organization's personnel identity caused by the enterprise split. This article takes a similar approach and corresponding measures to ensure the reliability of the study. First, the team of data analysts, in addition to the researchers involved in the survey, also invited peer experts to review the research process and results with a view to enhancing confidence in the reliability of the research conclusions. Second, the researchers of this in-depth interview data analysis carefully analyzed and sorted the data. Third, from the beginning of the establishment of the framework discussion to the acquisition of the final in-depth interview information and data, more researchers participated. Among them, although two researchers did not participate in the in-depth interview, the data cluster analysis is more professional, so during the spindle coding, the two researchers were asked for criticism and suggestions for data collection and analysis, so that they could analyze the collected information from an objective standpoint.

### 3.4. Open Coding

After confirming the method of data analysis above, openly code the interview data. The process of open coding is to analyze the interview data word by word, extract the important content of the interview data, and conceptualize the key content. The specific open code is shown in Table 1.

### 3.5. Open Coding Principal Component Factor Analysis

This survey divides the constraints of the development of rural tourism into 46 evaluation factors such as housing subsidies and division of property rights. The questionnaire survey combines the above index system with Likert's five-point scale method. The score of each index is 5–1 point from the options of strongly agree, agree, uncertain, disagree, and strongly disagree. High means that the approval of each element is higher. From the calculation results, the average score of 46 rural tourism development impact factors is between 3.066 and 4.569, the standard deviation is between 0.497 and 1.063, and the median is mainly concentrated in the two numbers, 4 and 3. In general, the average score is high, the standard deviation is not large, and the degree of dispersion of the score is more concentrated. The reason for the high average value is that with the rapid development of rural tourism, the extensive development mode with “quantity” as the development goal has gradually attracted everyone's attention and recognition. In order to further confirm whether there is a correlation between the 46 variables, this article uses the correlate command of Stata15.0 measurement software for processing and finds that there are many variables that have a very strong correlation, and some even exceed 90%, which indicates that there is a relationship between variables. With a considerable amount of information overlapping, it is very necessary for us to perform principal component analysis to integrate many initial variables into a few principal component variables that are not related to each other. From the perspective of 46 principal components, only the eigenvalues of the first three principal components are greater than 1, and the variance contribution rate of the first three principal components reaches 0.919, which basically meets our original intention of principal component analysis, but in order to further deepen and expand the principal component analysis and to study the related issues more thoroughly, we now cut into factor analysis. Factor analysis is an extension of principal component analysis. Its basic principle is to combine multiple variables with certain correlations into a few factors, so as to study how a set of measured indicators with intricate relationships is affected by a few internal factors. Independent factors dominate, so it belongs to a common statistical method for multidimensional analysis of dimensionality reduction problems. The measurement results are shown in Table 2.

From Table 2, we can see that a total of 1367 samples participated in the analysis and three retention factors were extracted. The chi-square value of the model LR test (LR test: independent vs. saturated: chi2 (1081) = 1.7*e* + 04) was 1.7*e* + 04, *P* value (Prob > chi2) is 0.001, and the model is very significant. The variable column represents the variable name, and the three columns, Factor1, Factor2, and Factor3, respectively, describe the degree of interpretation of the first three main factors extracted (generally, the system automatically selects feature values greater than 1) for each variable. The uniqueness column represents the part of the variable that has not been extracted and explained by the first three main factors. It can be found that the loss of information is relatively small when other main factors are discarded.

To better explain and name the variables, this paper rotates the factor structure and uses the predict command to obtain the factor score. The concept of factor score is a linear situation composed of each factor by normalizing each variable to mean equal to 0 and variance equal to 1 and then weighted by factor analysis coefficients. The factor's variance contribution rate is the weighted sum of the factors, and the comprehensive score of the factor for each sample can be obtained, as shown in Table 3. Before conducting the principal component factor analysis, standardize the constructed rural tourism industry sustainable development index variables through the measurement software Stata and use the KMO value to test whether the original variables are suitable for principal component factor analysis. The KMO value is 0.9615, ranging from 0.5 to 1.0; it is very suitable for factor analysis.

It can be seen from Table 4 that the cumulative contribution rate of the three principal component factors is 91.9% > 60%, and the principal component factor analysis can be performed completely. Three principal component factors (Factor1 (*F*_1_), Factor2 (*F*_2_), and Factor3 (*F*_3_)) are selected for comprehensive evaluation. From the principal component factor analysis coefficient, it can be seen that *F*_1_ reflects villagers' independent operation in policy incentives, distribution methods, and evaluation criteria which is difficult to achieve scale and income, villagers' enthusiasm for participating in rural tourism and villagers' shares in rural tourism, travel time and cost of tourism principles, image promotion of government information on tourism information, tourism logos of tourism motivation, the talent effect of the trust mechanism, the risk of resource integration and the comparison of income and the involvement of enterprises, and the acquisition of resources by enterprises. Different stakeholders consider different perspectives of benefits and costs, which leads to the existence of conflicts. The protection of innovation by property rights in the role and the division of property rights are too serious. 26 factors are related, mainly reflecting the sustainable development of rural tourism under the driving force of government, labor, capital, location, products, and other factors of rural tourism development. Influencing factors: *F*_2_ reflects housing subsidies in policy incentives, pollution of structural barriers that is difficult to cure, income from evaluation standards which determines the enthusiasm of villagers to participate in rural tourism, traffic conditions and tourism costs in tourism principles, local government in tourism information timely feedback on rural tourism destination information, tourism management, whether the tourism environment is comfortable and leisure, tourism motivation, tourism trust, creativity of tourism resources, integration of rural cultural resources, resource acquisition, resource control by the village leaders, and the scale of capital restrictions in resource barriers. The conflicts of interest determine the villagers' attitudes, the location conditions in the competition conditions that are related to the development of related industries, the protection of innovative products in the role of property rights, and other 22 factors, which mainly reflect the essence of rural tourism industry development and the sustainable development of rural tourism under the constraints. Influencing factors: *F*_3_ reflects 24 factors such as policy incentives, distribution methods, structural obstacles, evaluation criteria, tourism principles, tourism information, tourism management, tourism environment, tourism motivation, tourism trust, and trust of tourists in the main body of the relevant tourism destination, mainly embodying the influence factors of rural tourism development's customary thinking of various stakeholders on the sustainable development of rural tourism. From this, the weight coefficients of each index are further obtained, and the formula for calculating the comprehensive evaluation index of the sustainable development index of rural tourism is constructed:

(1) $$\begin{array}{c} F=0.326F_{1}+0.306F_{2}+0.287F_{3}. \end{array}$$

In the comprehensive evaluation model of principal component factors, the variance contribution rate of *F*_1_ reached 32.57%, indicating that the internal driving force of factors such as the role of government, labor, capital, location, and products in the development of rural tourism is strongly related to *F*, and it reflects 26 types. Among the factors, villagers have a fair distribution method, it is more difficult for villagers to operate independently, it is more difficult for the government to promote rural tourism destinations, it is more difficult for enterprises to obtain tourism resources and stimulate village democratic participation, and there are lower profit margins and scarcity of tourism service talents. The protection coefficient of the product is the highest. It can support enterprises through government policies, the government and enterprises encourage villagers to actively participate, and the local government promotes more; the variance contribution rate of *F*_2_ reaches 30.62%, indicating that rural tourism development is affected by factors of tourism resources (such as housing and land restrictions) and the nature of rural tourism development (such as the comfort, safety, and trust brought by the combination of nature and culture), which is highly relevant to *F*. Among the 22 factors reflected in it, pollution of rural tourism destinations, villagers' income, whether the government provides regulated services and constraints on tourists, the improvement of infrastructure, the creation of a safe atmosphere, the innovation of tourism products, and the location condition coefficient are the highest, meaning that rural tourism development is subject to transportation constraints and tourism products. Development and income from participating in village tourism development with villagers are mainly through improving infrastructure, designing rural tourism products according to consumer needs, increasing government assistance to rural tourism services, and improving villagers' income. The *F*_3_ variance contribution rate is 28.71%, indicating that rural tourism development is subject to government policies and evaluation criteria for villagers' participation in rural tourism development and whether tourists' travel is strongly related to *F*. Among the 24 factors reflected in it, a large number of zombies exist: pollution in rural tourist sites is difficult to control, villagers have a higher proportion of migrant workers, the control of villagers' free time to join rural tourism and the improvement of the environment, the amount of time spent traveling, the evaluation of the tourist environment and other tourists, and the behavior of the person in charge of the village collective organization. The involvement of enterprises and whether the village collective organization has the highest coefficient of control over resources mean that the development of rural tourism is subject to the vitality of rural tourism development, the participation of villagers, the reputation of the tourist destination, and the head of the village collective organization and the enterprise.

In the mean analysis, the rural tourism environment, the motivating factors of tourism, the creation of a safe atmosphere in rural tourism destinations, the attitudes of villagers, the supervision of rural tourism management and restrictions on tourists, the innovation and protection of tourism products, the government's publicity of tourist destinations, the location conditions of competition conditions, the development of other industries, and the convenience of transportation are all scored above 4 points, indicating that experts, tourists, villagers, entrepreneurs, village collective economic leaders, etc. participating in the questionnaire recognize these factors higher, which have a greater impact on the sustainable development of rural tourism. In the principal component factor analysis, the variance contribution rate of *F*_1_ is higher, indicating that among the factors affecting the sustainable development of rural tourism, the villagers tend to demand the villagers' fair distribution method and the villagers' independent operation. It is more difficult to introduce other social capital, strengthen the government's promotion of rural tourism destinations, village collective economic organizations to assist enterprises to obtain tourism resources and stimulate village democratic participation, increase profit margins, introduce tourism service talents, and increase rural tourism innovation products.

### 3.6. Spindle Coding

From the index design to the extraction of principal component analysis factors, the analysis idea is to extract the components by summarizing the conceptualized content and its relevance and the correlation between different conceptualized content to form a generalized main axis factor, which is the main axis coding. Combine the conceptualization formed by the open coding in Table 2, realize the categorization of conceptualized information according to the principal component factor analysis, and summarize the information logical relationship of categorized coding to extract three main categories, namely, social norms, value structure, and resource allocation. The main categories and their corresponding open codes are shown in Table 4.

After the formation of the main category to the final selective coding stage, its role is to clarify the relationship between the main category and the core category, to reach the theoretical saturation and form a conceptual model, in-depth interviews, index selection, and main component factors. Based on the combination of extraction (that is, the combination of open coding and spindle coding), a structural model of factors affecting the sustainable development of rural tourism is constructed, as shown in Figure 1.

### 3.7. Research Findings

Data analysis after in-depth interviews found that the sustainable development of rural tourism faces three major pressures: social norms, value structure, and resource allocation. In the absence of an effective coordination mechanism under the three major pressures, rural tourism development seems to be more inclined to “short and fast” and “conventional” production methods, thus restricting the growth of rural tourism.

### 3.8. Social Normative Pressure

The interview data show that the sustainable development of the rural tourism industry is constrained by social normative pressure. First of all, the current production and lifestyle of the villagers still dominate the modern rural production and lifestyle. The villagers are always engaged as foreign workers or independently operating small-scale farmhouses. Fei [40] stated that China's rural areas are typical rural villages, with little change, stable culture, and few new problems. They do not want their lifestyle and rhythm to be disrupted. Second, villagers are faced with conflicts of interest with various stakeholders. Whether the interest acquisition of the transfer of resources and the value of the benefits match the value of the resources is directly related to a series of factors such as the trust mechanism, distribution methods, and evaluation standards. They think more about short-term profits. Third, how to deal with the issues of ethics and legal norms, the lack of protection of property rights, the mutual duplication of tourism products, and the severe division of property rights has caused the resources to be more scattered, which has restricted the development of rural tourism to varying degrees. In short, in the existing rural tourism, villagers and other stakeholders have tended to obtain economic income faster in the existing market system, which has imposed social normative pressure on long-term tourism development planning. Under such pressure, villagers and other stakeholders are more likely to choose extensive rural tourism development methods in order to obtain more stable income support.

### 3.9. Value Structural Pressure

The interview data show that the development of rural tourism is also constrained by structural pressure on value. This structural pressure on value is mainly reflected in the following three aspects: first, the tourism value contained in the tourism resources held by the villagers. First, the villagers are not clear about the impact of their value on rural tourism and their attitudes on rural tourism: just as a farmer said, “Labor has also become part of the development of rural tourism? This is not understood.” Second, the villagers believe that the satisfaction of rural tourists is not determined by him and has little to do with him. Second, the evaluation criteria of tourists on the value of tourism products: the evaluation of tourists on tourist destinations is a combination of multiple factors, and the combination of multiple factors is difficult to satisfy all. As a result, tourism development products are copied more seriously, such as environmental construction and copy of management system. Third, the amount of tourists and income are used to measure the quality of rural tourism development. For example, some regions use ticket income to obtain a large amount of short-term benefits. These development methods, which are consistent with conventional and conservative values, comparative evaluation standards, and production standards in accordance with “manufacturing,” have become the shared concepts and ways of thinking of rural tourism development. Also, this kind of thinking is unconsciously accepted by the majority of stakeholders, which restricts the continuation of the life cycle of the rural tourism industry.

### 3.10. Resource Allocation Pressure

In addition to social normative pressure and value structural pressure, the development of rural tourism is also facing resource allocation pressure. First of all, in rural economic development, it is widely recognized that agriculture is the main production method. For food subsidies, even the barren land for many years has recently been reclaimed and planted, and it is more difficult to levy construction land just needed for tourism. Second, the implementation of the rural revitalization strategy, the introduction of a large number of rural tourism projects, the suitability of the local ecology, the richness of the tourism culture, and the competitive advantage are all lacking in consideration. Third, the obstacles to resource integration, resource acquisition, and resource development have, to a certain extent, led to the formation of dead projects and the waste of resources. Moreover, the widespread existence of such resource allocation pressure has broken or induced rural tourism development to lack the depth and length of development, thus restricting the long-term strategic development of rural tourism.

## 4. Conclusions, Limitations, and Future Research

The main purpose of this article is to explore the constraints and countermeasures for the practical problems facing the sustainable operation of rural tourism under the great development of rural tourism. Through in-depth interviews with 190 rural tourism stakeholders in the three provinces of Henan, Hunan, and Guangdong, the study found that the development of rural tourism continues to be constrained by three kinds of pressures: (1) social normative pressures, including those that are conducive to conventional agriculture, contradictions such as policy incentives for the development of a household-to-household, lack of power and responsibility mechanisms applicable to the sustainable development of rural tourism, and conflicts of interest among the main bodies of the sustainable development of rural tourism; (2) value structure pressure, including differences in the evaluation of the value of tourism resources, the destruction of the integrity mechanism, the complexity of the management system, and the formation of criteria for evaluating the development of tourism destinations based on price and revenue; (3) pressure on resource allocation, including policy-oriented investment practices, relying on government “blood transfusion” assistance, and consumer demand for tourism diversification and specialization. In addition, under the three pressures, the various interest subjects are able to achieve the desired utility for their own needs, and they are more inclined to obtain instant benefits, which hinders the continuous development of the rural tourism industry. This study has several limitations. The measurements of the limitations of rural tourism destinations are investigated. China is a multiethnic country, and a small sample might create a social desirability bias [41, 42]. The online survey response rate was relatively low; thus, there was a nonresponse bias. Individuals who may have different opinions were unable or unwilling to participate.

Future research will confirm the impact of stakeholder demand-driven issues on rural tourism destinations. There may be many variables in the demand drivers of stakeholders. The study of these variables is helpful to the sustainable development of rural tourism destinations. Qualitative research may reveal the attitude of stakeholders towards rural tourism destinations and their feelings about development. Future research can control different driving factors to further promote research. Other intermediary factors can also be considered, such as emotional energy factors, to regulate the sustainable development behavior of stakeholders.

## Figures and Tables

**Figure 1:** The analysis of the obstacles to the growth of rural tourism.

**Table 1:** Examples of open coding processes.

Interview crowd	Interview materials (partial citations)	Process	
		Conceptualize	Category
Community residents	“Now the government encourages us to plant fields, an acre of grain directly to supplement 105 yuan, two-season rice subsidy 170 yuan. In addition to subsidies for growing rice, we have subsidies for growing wheat, corn, and other crops. Development tourism says to plant other flowers and grasses, but these are not subsidized.	Production subsidies are better	Policy incentives
	“Now the government is encouraging us to move to the city and live in a one-to-one payout to give us housing subsidies. It requires us to contract the fields to the enterprise for special operation. But I'm a farmer, and I only do farm work.”	Unreasonable housing subsidy	
	......	......	

Tourists	“When the weather is nice, we usually use the weekend to go for a walk around the countryside and relax. If it's a long vacation, little consideration is given to rural tourism.	Time, traffic constraints	Travel motivation
	“Roads are not easy to walk, not easy to drive (note: rural tourist destinations), we generally do not go.”		
	“It's a real country tour that evokes memories of our childhood.	Lack of character	
	“Now a lot of country tourism is done the same, no taste, go once and do not want to come a second time.”		
	......	......	

Head of collective economic organization	“It's too difficult for farmers to organize now, and once economic interests are involved, it's hard to adjust.”	Managers are less convinced	Trust mechanisms
	“The election of the head of a collective economic organization, whoever is elected, is more or less discussed.”		Structured barriers
	“I've tried to take the lead in dealing with these things, but I've always been doubted, and it's hard for me to do it.”		
	“The income has not been significantly increased, and it is difficult to achieve the participation of all the villagers.”	The real problem of risk and income	
	“Farmers earn their money through hard work. They do not want to use their money for risky investment, so the villagers to invest in shares, together to build some infrastructure problems, is difficult.”		
	......	......	

Local government workers	“We do a lot of work on environmental governance, such as funding and sanitation worker in situ, but when it comes to the peak tourist season, there are a lot of environmental pollution problems that we cannot control, such as some tourists' habitual behavior which we cannot correct.”	Environmental change requires process	Behavioral practices
	“Before we could develop rural tourism, our villagers had to build houses with wood, which led to the cutting down of many ancient trees.”	The destruction of the original ecology of plants and animals	
	“Some tourists do not pay much attention, resulting in some damage to the original ecology of plants and animals.”		
	“Some local villagers run farmhouses, some waste water discharges are not paid much attention, although many reminders, but the effect is not very good.”		
	......	......	

Head of rural tourism enterprises	“In recent years, there have been at least 100,000 rural tourism developments throughout the country, and special towns, pastoral complexes, and special villages have blossomed everywhere. High-density rural tourism development mode is not conducive to the healthy development of rural tourism.”	The same type of tourism products has a greater impact	Competitor threats
	“There has to be an influential campaign to do the publicity, or it's likely to go to dry.”		
	“New travel products are replaced quickly, and the conversion costs are high if we want to do it.”	New types of tourism products are emerging	
	......	......	

**Table 2:** Main categories formed by spindle coding.

Main category	Corresponding concepts and subcategories	The meaning of category
Social norms	Distribution mode Structured barriers Evaluation criteria Trust mechanism Conflicts of interest Property rights	Fair and equitable distribution is conducive to stimulate the enthusiasm of villagers to participate in rural tourism, villagers' inertial lifestyle and evaluation criteria have certain structural obstacles to the development of rural tourism, and for the trust mechanism between people, conflicts of interest and the norms of property rights system, etc. have different regular manifestations.

Value structure	Tourism principles Tourism information Tourism management Tourism environment Tourism motivation Tourism trust Tourism resources	The determination of the value of rural tourism products depends on transportation, time, cost, information, management, trust, tourism resources, and motivation to initiate tourism activities, and they together constitute the brand value structure of rural tourism.

Resource allocation	Policy incentives Resource integration Resource access Resource barriers Competitive conditions	Encouraging the development of rural tourism is conducive to the rapid development of rural tourism, but the integration of rural tourism resources, difficult access and resource utilization obstacles, tourism products, location disadvantage, and related industries supporting the development of rural tourism are the bottleneck of sustainable development of rural tourism.

**Table 3:** Principal component factor analysis of sustainable development of rural tourism industry.

Principal component factor	Variance	Variance contribution rate	Total
Factor1 (*F*_1_)	15.308	0.326	0.326
Factor2 (*F*_2_)	14.393	0.306	0.632
Factor3 (*F*_3_)	13.493	0.287	0.919

**Table 4:** Basic situation of variable factor analysis of sustainable development of rural tourism industry.

Variable	Factor1	Factor2	Factor3	Uniqueness
A1	0.931	0.113	–0.083	0.113
A2	0.950	–0.187	0.024	0.062
A3	0.881	0.343	–0.077	0.101
A4	0.927	–0.170	–0.188	0.077
A5	0.861	0.126	0.364	0.110
A6	0.944	0.223	–0.009	0.060
A7	0.939	0.083	–0.202	0.071
A8	0.919	0.310	0.025	0.059
A9	0.927	–0.286	0.062	0.055
A10	0.907	0.220	0.049	0.126
A11	0.944	0.123	–0.115	0.081
A12	0.915	–0.142	0.281	0.064
A13	0.942	0.229	–0.014	0.059
A14	0.951	–0.135	–0.059	0.075
A15	0.950	–0.035	–0.205	0.055
A16	0.933	–0.262	0.112	0.048
A17	0.920	–0.191	0.185	0.084
A18	0.936	–0.204	0.169	0.055
A19	0.778	0.466	0.226	0.127
A20	0.884	0.166	0.237	0.135
A21	0.876	0.199	0.297	0.105
A22	0.930	–0.129	0.240	0.061
A23	0.947	–0.076	–0.026	0.096
A24	0.925	–0.160	0.241	0.061
A25	0.897	–0.058	0.319	0.091
A26	0.916	–0.209	0.255	0.053
A27	0.946	0.109	–0.128	0.077
A28	0.933	0.194	0.020	0.092
A29	0.936	0.132	–0.103	0.096
A30	0.928	–0.262	–0.076	0.065
A31	0.896	0.390	0.032	0.044
A32	0.913	0.149	–0.242	0.086
A33	0.936	0.173	0.101	0.084
A34	0.938	–0.002	–0.247	0.059
A35	0.946	0.040	–0.198	0.065
A36	0.943	–0.072	–0.214	0.060
A37	0.945	–0.154	–0.120	0.070
A38	0.936	0.113	0.039	0.110
A39	0.923	–0.157	–0.184	0.090
A40	0.945	0.042	–0.144	0.085
A41	0.920	–0.234	–0.104	0.089
A42	0.950	0.157	–0.090	0.064
A43	0.913	–0.301	0.033	0.076
A44	0.893	–0.235	0.109	0.135
A45	0.917	–0.233	–0.085	0.098
A46	0.922	–0.023	–0.167	0.121

## Data Availability

The data are available on request.
